The article "FKN/NR Signaling Pathway Regulates Hippocampal Inflammatory Responses: the Survival of Hippocampal Neurons in Diabetic Rats with Chronic Unpredictable Mild Stress" was published in 2022. Journal: Evid Based Complement Alternat Med.

# FKN/NR Signaling Pathway Regulates Hippocampal Inflammatory Responses: the Survival of Hippocampal Neurons in Diabetic Rats with Chronic Unpredictable Mild Stress

**DOI:** 10.1155/2022/8980627

**Published:** 2022-08-29

**Authors:** Zhuo Liu, Hongqing Zhao, Jian Liu, Yuanshan Han, Yuhong Wang

**Affiliations:** ^1^Affiliated Hospital of Hunan Academy of Traditional Chinese Medicine, Changsha, Hunan, China; ^2^Hunan University of Chinese Medicine, Science and Technology Innovation Center, Changsha, Hunan, China; ^3^First Affiliated Hospital of Hunan University of Traditional Chinese Medicine, Changsha, Hunan, China

## Abstract

**Aim:**

To investigate the mechanism via which FKN/CX3CR1 signaling abnormalities mediate N-methyl-D-aspartic acid receptor (NMDA) overexcitation-induced hippocampal neuronal injury in diabetic rats complicated with depression (DD).

**Methods:**

Sixty rats were randomly divided into 5 groups. The depression-like behaviors of the rats were evaluated by open field test and Morris water maze. The pathological changes of hippocampus in DD rats were observed by HE staining. The blood levels of inflammatory factors (IL-1*β*, TNF-*α*, and IL-6) and neurotransmitters (D-serine and glutamic acid) were determined by enzyme-linked immunosorbent assay (ELISA). The expressions of BDNF, A1 receptor (A1R), A2 receptor (A2R), A3 receptor (A3R), calmodulin dependent kinase II (CaMKII), CX3CR1, CX3CL1 (FKN), NR2A, and NR2B proteins were detected by immunohistochemistry and Western-blotting.

**Results:**

Compared with the normal control group, blood glucose level increased significantly and body weight decreased in T2DM group and T2DMC group. In addition, the number of spontaneous activities significantly decreased and the capability of learning and memory was attenuated in T2DMC group and Chronic Stress group. The blood levels of IL-1*β*, TNF-*α*, IL-6, glutamate (Glu), and D-serine significantly increased in each model group. After intervention with CX3CR1 antibody, the expressions of BDNF, CaMK II, A1R, and A3R increased and those of A2R, CX3CR1, FKN, NR2A, and NR2B decreased.

**Conclusion:**

In the diabetic state, the binding of FKN to CX3CR1 increases, which regulates a variety of adenosine receptors. When it exerts its effect on neurons, the overactivation of NR results in neuronal injury and causes depression.

## 1. Introduction

Diabetes is a metabolic disease characterized by high blood glucose levels [1]. The incidence of depression is as high as 10%–40% in patients with type 2 diabetes mellitus (T2DM) [2, 3]. The death risk increases by 1.5 times in patients with diabetes mellitus with depression (DD) [4]. Compared with nondiabetic patients, diabetic patients are nearly five times more likely to suffer from depression, and the recurrence rate is 8 times higher [5]. Obviously, diabetes and depression are highly comorbid [6]. As a highly recurrent and fatal condition, DD can directly affect the patients' quality of life and physical and mental health [7–9]. Therefore, it is important to prevent and treat DD based on its pathogenic mechanism.

The article "FKN/NR Signaling Pathway Regulates Hippocampal Inflammatory Responses: the Survival of Hippocampal Neurons in Diabetic Rats with Chronic Unpredictable Mild Stress" was published in 2022. Journal: Evid Based Complement Alternat Med.

However, few studies have explored the pathogenesis of DD, which mainly focused on the hippocampus, the key brain structure that is involved with learning and memory [10]. Research has shown that the hippocampal neurons in the rat DD models were arranged disorderly, the cells were vacuolated, and the blood-brain barrier was damaged [11]. Based on numerous experiments, we had established a stable and reliable animal DD model in our previous study, and further studies have shown that the hippocampal neurons (Ne) in DD rats experienced obvious apoptosis [12]. However, how the hippocampal neurons are damaged in DD has not been reported.

Fractalkine (FKN), a microglia activation chemokine specifically expressed in neurons and knockout of the FKN receptor CX3CR1, is predominantly expressed in microglia [13]. Studies suggest that increased FKN and CX3CR1 may cause a cross-talk between activated glial cells and neurons, playing an important role in the development of neuroinflammation in mice [14].

Application of FKN triggered a 53% reduction of the NMDA-induced neuronal calcium influx [15]. Previous studies have implicated inflammation in the brain for impairment of central nervous system (CNS) nerves, a known high-risk factor for diabetic encephalopathy [16].

It has been found that the fractalkine (FKN)/CX3CR1 signaling pathway regulates the transmission of information between hippocampal neurons, triggering a proinflammatory response and inducing depression [6].

Meanwhile, the presence of NMDA receptor-mediated responses in hippocampal CA1 neurons, a synaptic mechanism for hippocampal processing that may play important roles in hippocampus-dependent functions such as learning and memory [17].

Further research showed that the FKN/CX3CR1 signaling pathway induced the release of inflammatory factors including tumor necrosis factor-*α* (TNF-*α*), interferon-*γ* (IFN-*γ*), and interleukin-1*β* (IL-1*β*) *in vivo*. In streptozotocin-diabetic rat (STZ-rat), spatial learning impairments develop in parallel with a reduced expression of long-term potentiation (LTP) and enhanced expression of long-term depression (LTD) in the hippocampus, affected by NMDA receptor (NR) activation [18]. Recent study shows that NR plays a key role in chronic inflammation, learning and memory, behavioral cognition, and synaptic plasticity [19]. Furthermore, NR activation and hippocampal neuronal injury induced DD [12].

The article "FKN/NR Signaling Pathway Regulates Hippocampal Inflammatory Responses: the Survival of Hippocampal Neurons in Diabetic Rats with Chronic Unpredictable Mild Stress" was published in 2022. Journal: Evid Based Complement Alternat Med.

The relationship between inflammatory response with NR in the hippocampus and diabetes-related depression is not well understood. In this study, we investigated the role of FKN/CX3CR1 signaling pathway in hippocampal neuronal injury, in an attempt to further identify the pathogenesis of DD.

## 2. Materials and Methods

### 2.1. Experimental Animals

In total, 60 male Sprague-Dawley (SD) rats (male, weighing 180–220 g, of SPF grade, and production license no. SCXK 2009–0004) were purchased from the Hunan SJA Laboratory Animal Co., Ltd. (Hunan, China), and maintained in the SPF level barrier environmental facilities in the laboratory animal center of the First Affiliated Hospital of Hunan University of traditional Chinese Medicine. They were housed in an ambient room temperature (25 ± 2°C) and relative humidity (50 ± 5%), with a 12 h dark-light cycle and unrestricted diet for five days, which were used to adapt rats to the environment.

This study was approved by the Experimental Animal Ethics Committee of Hunan University of Chinese Medicine (NO2019070611), and the study protocol met the national requirements for medical experimental animals.

### 2.2. Experimental Design

Sixty rats were split up into five parallel groups randomly (*n* = 12 in each group). Rats were divided into two parts: 24 were randomly divided into normal group and Chronic Stress (CS) group, and 36 were used to establish diabetes models. Diabetes models were randomly divided into type 2 diabetes mellitus (T2DM) group, T2DM + Chronic Stress (T2DMC) group, and T2DM + Chronic Stress + CX3CR1 (T2DMCC) group, with 12 rats, respectively.

The diabetes models were established as follows: the rats were fed a lipid emulsion containing 10% cholesterol, 0.2% propylthiouracil, 20% lard, 2% sodium cholate, 20% Tween-80, and 20% propylene glycol at a dose of 10 mL/(kg·d). After 14 consecutive days of intragastric administration, the rats were injected with streptozotocin (STZ) (38 mg/kg) via the tail vein, and the fasting blood glucose level was measured 72 hours after STZ injection. Rats with a fasting blood glucose level ≥16 mmol/L were randomly divided into T2DM group, T2DMC group, and T2DMCC group. For the T2DMCC group, intraperitoneal injection of CX3CR1 neutral antibody (80 *μ*g/(kg·d)) was initiated in the Chronic Stress models once a day. Other groups were injected with saline.

Thereafter, rats in the normal group and the T2DM group were normally fed, and the Chronic Stress group and the T2DMC group continued to be subjected to chronic unpredictable mild stress for 28 days. The stressors included bath in cold water at 4°C, bath in hot water at 45°C, electric shock, reversed light-dark cycle, and tilting of home cage. One stressor was randomly applied on a daily basis, and the same stressor was not applied consecutively. All rats were tested for behaviors upon the completion of modeling. After the test was completed, blood samples were collected from the abdominal aorta. The hippocampus was harvested and cryopreserved in liquid nitrogen in 6 rats in each group; for the remaining 6 rats, the brain tissue was harvested after polyformaldehyde perfusion and then fixed in a formaldehyde solution (Figure 1). For the T2DMCC group, intraperitoneal injection of CX3CR1 neutral antibody (80 *μ*g/(kg·d)) was initiated in the Chronic Stress models.

The article "FKN/NR Signaling Pathway Regulates Hippocampal Inflammatory Responses: the Survival of Hippocampal Neurons in Diabetic Rats with Chronic Unpredictable Mild Stress" was published in 2022. Journal: Evid Based Complement Alternat Med.

### 2.3. Drugs and Raw Materials

The raw materials and drugs included cholesterol, propylthiouracil, lard, Tween 80, propylene glycol, and streptozotocin (Beijing Solarbio Science and Technology Co., Ltd., China). Rabbit anti-polyclonal CX3CR1, FKN, was purchased from Abcam, UK; rabbit anti-polyclonal NR2A and NR2B antibodies were purchased from CST, USA, while GAPDH was purchased from Proteintech, USA. Streptozotocin and dexamethasone (Dex) were purchased from Saint Louis, MO, USA. IL-1*β*, interleukin-6 (IL-6), interleukin-8 (IL-8), and TNF-*α* enzyme-linked immunosorbent assay (ELISA) kits were purchased from Jingtian Biological Technology Limited Company, Shanghai, China. Cholesterol (CT), corticosterone (CORT), corticotropin (ACTH), and hypothalamic corticotropin-releasing hormone (CRH) ELISA kits were from R&D Systems, Minnesota, USA. Dulbecco's modified eagle medium/nutrient mixture F-12 medium, B-27 culture additive (GIBCO), and fetal bovine serum were from HyClone Corporation, Logan City, Utah, United States. Triglycerides (TG), high density lipoprotein cholesterol (HLD-C), and low density lipoprotein cholesterol (LDL-C) ELISA kits were from Beijing Zhongsheng Biological Technology Limited Company, Beijing, China.

### 2.4. Behavioral Tests

#### 2.4.1. Open Field Test (OFT)

Rats were placed in a black open field box sized 80 cm × 80 cm × 40 cm with 25 wells at the bottom. Each time, they were placed from the same corner. After the rats were acclimated for 1 min, the number of horizontal movements (with four paws in the grids) and the vertical standing (with two front paws lifted) within 3 min were recorded.

#### 2.4.2. Morris Water Maze (MWM)

The Morris water maze (MWM) test lasted 5 days (place navigation training for 4 days and test on the 5th day). During the place navigation test, a hidden platform was located under the water's surface. The rats were placed in the maze, and the time spent on finding the hidden platform (the latent period) was recorded. The time limit was 60 s, and the time exceeding 60 s was recorded as 60 s. In addition, after the platform was removed, the time of rats spent on the target quadrant (target quadrant memory time) within 60 s was recorded.

The article "FKN/NR Signaling Pathway Regulates Hippocampal Inflammatory Responses: the Survival of Hippocampal Neurons in Diabetic Rats with Chronic Unpredictable Mild Stress" was published in 2022. Journal: Evid Based Complement Alternat Med.

#### 2.4.3. Forced Swim Test (FST)

Forced swim test was performed for assessing giving-up-like depression behavior. Briefly, this test needs a circular fibreglass pool containing warm water (25 ± 1°C). And, in this experiment, immobility time was determined by the time in which a rat stopped struggling. Moreover, moving slowly to remain floating in the water was seen as immobility.

### 2.5. Blood Glucose Measurement

Animals were fasted for food, but not for water for 8h. Blood was collected from the tail vein and glucose level was measured by a blood glucose meter.

### 2.6. HE Staining

The brain tissue fixed in the formaldehyde solution was conventionally dehydrated, embedded in paraffin, and cut into 5 *μ*m thick serial sections. The specimens were fixed for 24 h, immersed in 0.01 mol/L PBS for 12 h, dehydrated after hematoxylin-eosin staining, sealed with neutral gum, and then observed under an optical microscope. Photographs were taken to analyze the hippocampal injury in each group.

### 2.7. Detection of Insulin and Glycosylated Hemoglobin

When collecting blood from abdominal aorta, anticoagulant tube was used to collect blood, and the supernatant was collected after centrifugation and stored at −80°C. Operate in strict accordance with the kit when testing.

### 2.8. Detection of Glu, D-serine, and Inflammatory Factors in Plasma

When collecting blood from abdominal aorta, anticoagulant tube was used to collect blood, and the supernatant was collected after centrifugation and stored at −80°C. The test shall be carried out in strict accordance with the instructions of ELISA kit. Specific indicators include glutamic acid (Glu), serine (D-serine), interleukin-1*β* (Interleukin-1, IL-1*β*), and tumor necrosis factor-*α* (tumor necrosis factor-*α*, TNF-*α*).

### 2.9. Detection of Monoamine Neurotransmitters

HPLC-EDU chromatographic conditions: chromatographic column: 150 × 2.1 mm, 3 *μ*m Hypersil BDS C18 column; mobile phase: A: containing 90 mM sodium dihydrogen phosphate monohydrate, 50 mm citric acid monohydrate, and 1.7 mm sodium octane sulfonate 50 *μ*m EDTA mixture; B: methanol; A : B (93 : 7); flow rate: 0.2 ml/min; column temperature: 30°C; sample size: 20 *μ*L.

Sample handling: the cryopreserved hippocampus was weighed precisely, and 0.01 M perchloric acid solution containing 0.03 mm EDTA and 10 mg/L internal standard DHBA were added to prepare a 1 : 3 tissue homogenate. It was centrifuged at 13000 r/min at 4°C for 10 min. After standing, the supernatant was carefully collected.

The article "FKN/NR Signaling Pathway Regulates Hippocampal Inflammatory Responses: the Survival of Hippocampal Neurons in Diabetic Rats with Chronic Unpredictable Mild Stress" was published in 2022. Journal: Evid Based Complement Alternat Med.

Standard product configuration: dissolve 1 mg of NA, DA, and 5-HT standards, respectively, in 1 mL of 0.01 M perchloric acid solution containing internal standard, dilute them into 6 concentrations in equal proportion of 0.5 times, and calculate the standard curve (see Table 1).

### 2.10. Immunohistochemical Examinations of A1R, A2R, A3R, CX3CR1, FKN, NR2A, and NR2B, CaMKII, and BDNF

The whole brain tissue was fixed, embedded in paraffin, and sliced. The sections were dehydrated through graded ethanol (75%, 95%, and 100%). Following antigen retrieval, sheep serum confining liquid was added at 37°C for 30 min. After serum was removed, A1R, A2R, A3R, CaMKII, BDNF, CX3CR1, FKN, NR2A, and NR2B primary antibodies were added and incubated overnight at 4°C. The sections were then washed with PBS three times and incubated with the secondary antibody for 10 min with the immunoreaction enhancer solution for 10 min. Then, the sections were rinsed, stained with DAB, counterstained with hematoxylin, dehydrated through graded ethanol, and sealed. The immunohistochemical sections were photographed at a high magnification (×400), and the integrated optical density (IOD) was analyzed using Image-Pro Plus software.

### 2.11. Western-Blotting

The hippocampus tissue was added with 1% PMSF cell lysate containing protease inhibitor, homogenized, and centrifuged at 12,000 r/min at 4°C for 5 min, and the supernatant was collected. The concentration of the protein samples was determined by a nucleic acid protein concentration meter. The supernatant was diluted to a target loading concentration of 200 *μ*g/10 *μ*L using PBS; 20 *μ*L of the diluted sample was placed into an EP tube, to which 5 *μ*L of 5 × loading buffer was added. After mixing, they were denatured in a PCR instrument at 100°C for 5 min. The same amount of protein samples was loaded, electrophoresed, and transferred to a PVDF membrane. The membrane was immersed in skim milk powder for 1 h and washed with TBST 3 times. It was incubated overnight at 4°C with A1R (1 : 1000), A2R (1 : 1000), A3R (1 : 1000), CaMKII (1 : 1000), BDNF (1 : 1000), CX3CR1 (1 : 1000), FKN (1 : 3000), NR2A (1 : 1000), NR2B (1 : 1000), and GAPDH (1 : 5000) primary antibody dilutions, respectively. After the secondary antibodies were added, the mixture was incubated at room temperature for 1 h. Autoradiography was performed using the ECL chemiluminescent substrate. The gray-scale values were calculated with the ImageJ software using the following formula: relative expression level of the target protein = gray value of target protein/gray value of internal reference.

The article "FKN/NR Signaling Pathway Regulates Hippocampal Inflammatory Responses: the Survival of Hippocampal Neurons in Diabetic Rats with Chronic Unpredictable Mild Stress" was published in 2022. Journal: Evid Based Complement Alternat Med.

### 2.12. *In vivo* Experiment

#### 2.12.1. Expression of CX3CR1, FKN, NR2A, and NR2B Proteins in the Microglia

Each culture plate well was fixed for 30 min at 37°C with 4% paraformaldehyde and then permeabilization for 15 min with 0.25% triton-100 and blocking 30 min using 5% bovine albumin.

In each well, *β*-Tubulin polyclonal antibodies 50 *μ*l (1 : 100), CX3CR1 (1 : 1000), FKN (1 : 1000), NR2A (1 : 1000), and NR2B (1 : 1000) primary antibodies were added and incubated overnight at 4°C. The wells were then washed with PBS three times and incubated with the secondary antibody for 10 min and incubated with the fluorescein 5-isothiocyanate for 30 min at 37°C. Thereafter, 4′, 6-diamidino-2-phenylindole (DAPI) (1 : 800) was added for 15 min incubation. Then, plates were having 50 *μ*l phosphate buffer saline to allow fluorescence observation and high content analysis (HCS).

### 2.13. Statistical Analysis

Statistical analysis was performed using the SPSS 23.0 software. The measurement data are expressed as mean ± SEM. Each indicator was tested by one-way analysis of variance (ANVOA), LSD test, and two-sided test.

## 3. Results

### 3.1. DD Rats Exhibit an Abnormal Body Weight, Blood Glucose Level, and Depressive-like Behavior

As shown in Figure 2(a), SD rats were given high-fat diet for 2 weeks, then injected with STZ, and followed by subjected Chronic Stress for 21 days to establish the diabetes-related depression model. After modeling, we found that DD reduce the desire to learn and explore, impairing memory. However, CX3CR1 neutral antibody treatment restored normal behavior and functioning of DD, and DD modeling obviously reduced the crossing scores and rearing scores in the open field test and also significantly increased the immobility time of DD rats in the forced swimming test (Figures 2(b) and 2(e)). Furthermore, as shown in Figures 2(c) and 2(d), there was a significance difference in body weight between groups, reflectively of glucose underutilization. These results indicated that the rat model of DD was successfully established and the DD rats exhibit depressive-like behavior, together with abnormal body weight and blood glucose. Blocker group revers the pathophysiology.

### 3.2. DD Aggravates Insulin and Glycosylated Hemoglobin Content

The plasma insulin in diabetes mellitus and depression group was significantly lower than that in the normal group (*P* < 0.01), and the glycosylated hemoglobin content increased significantly (*P* < 0.01), suggesting that the diabetic depression model had been successfully established (Figure 3). Blocker treatment regresses this pathophysiology across the group.

The article "FKN/NR Signaling Pathway Regulates Hippocampal Inflammatory Responses: the Survival of Hippocampal Neurons in Diabetic Rats with Chronic Unpredictable Mild Stress" was published in 2022. Journal: Evid Based Complement Alternat Med.

### 3.3. DD Increases the Expression of TNF-*α*, IL-1B, and IL-6 Proinflammatory Factors in the Hippocampus

As shown in Figure 4(a), compared with the normal group, there was a significant increase in TNF-*α*, IL-1B, and IL-6 in the hippocampus of diabetes, depression, and DD group (*P* < 0.01). However, TNF-*α*, IL-1B, and IL-6 secretion in DD group was significantly enhanced than that in depression and diabetes group (*P* < 0.05, *P* < 0.01); CX3CR1 blocker treatment of DD group significantly reduced the levels of TNF-*α*, IL-1B, and IL-6 in hippocampus of all groups (*P* < 0.05, *P* < 0.01). CX3CR1 blocker modulates undesirable inflammatory excesses in these tissues.

### 3.4. DD Increases the Expression of Glutamic Acid (Glu) and D-serine in the Hippocampus

As shown in Figure 4, compared with the normal group, there was a significant increase in Glu and D-serine levels in the hippocampus of diabetes, depression, and DD group (*P* < 0.01). However, Glu and D-serine levels in DD group were significantly enhanced than those in depression and diabetes group (*P* < 0.05, *P* < 0.01); CX3CR1 blocker treatment of DD group significantly reduced the levels of Glu and D-serine in hippocampus all group (*P* < 0.05, *P* < 0.01). CX3CR1 blocker modulates undesirable inflammatory excesses in these tissues.

### 3.5. DD Regulates the Monoamine Neurotransmitters in Hippocampus

Depression levels are reflected in the amount of DA, 5-HT, and NA in hippocampus. As shown in Figure 5, the contents of DA and 5-HT in hippocampus of diabetic rats, depression, and DD were significantly decreased (*P* < 0.05 or *P* < 0.01), and the content of NA increased significantly (*P* < 0.01). Therefore, even though diabetes, depression, and DD regulate secretion of DA, 5-HT, and NA, CX3CR1 blocker treatment modulates the secretion of the three monoamine neurotransmitters in DD rats.

### 3.6. Findings of HE Staining

The hippocampal neurons in normal rats had regular morphology and orderly arrangement, along with uniform chromatin structure and normal neuronal gaps. The hippocampal neurons in the model groups showed different degrees of cell swelling, nuclear pyknosis, deep cytoplasmic staining, disordered arrangement, and elongated gaps, especially in the T2DMC group. The hippocampal neurons in the T2DMCC group recovered markedly (Figure 6).

### 3.7. Immunohistochemical Findings of FKN/NR-Related Molecules

Microglia activation induced by neuroinflammation damages hippocampal neurons and high levels of inflammatory factors such as TNF-*α*. It can promote the release of chemokines and lead to the abnormal expression of FKN receptor CX3CR1 to mediate the occurrence of neuroinflammation [20]. CX3CR1 antibodies are potent repressors of NR activity and together downregulate both AR and NR. In addition, CX3CR1 and NR upregulate transcription of inflammation, which further damages the hippocampus. As shown in Figures 7(a) and 7(c), compared with the normal control group, the model groups of A1R, A3R, and A2R expressions in the hippocampus had significantly decreased. The expressions of A1R and A3R increased but A2R decreased in the T2DMCC group.

The article "FKN/NR Signaling Pathway Regulates Hippocampal Inflammatory Responses: the Survival of Hippocampal Neurons in Diabetic Rats with Chronic Unpredictable Mild Stress" was published in 2022. Journal: Evid Based Complement Alternat Med.

Compared with the normal control group, the number of BDNF and CaMKII immunoreactive cells in the hippocampus of the T2DM group and the T2DMC group significantly decreased (*P* < 0.05). In contrast, the expressions of these markers increased in the T2DMCC group, and the positive expression was obvious.

Compared with the normal group, the number of CX3CR1 and FKN immunoreactive cells significantly increased in the hippocampus of the T2DM group and the T2DMC group (*P* < 0.05) and significantly decreased in the T2DMCC group (*P* < 0.01).

Compared with the normal group, the expression levels of NR2A and NR2B significantly increased in the model groups and significantly decreased in the T2DMCC group (*P* < 0.01, *P* < 0.05) (Figures 7(a) and 7(c)).

### 3.8. Western-Blotting Results of FKN/NR-Related Molecules

As shown in Figures 7(b) and 7(d), compared with the normal control group, the model groups had significantly decreased protein expressions of A1R and A3R and increased protein expression of A3R. In the T2DMC group, the decrease in the protein expressions of A1R and A3R was even more obvious than in the Chronic Stress group and the T2DM group.

Compared with the normal control group, the model groups showed a significant decrease in BDNF and CaMK II, while the reduction in BDNF and CaMK II in the T2DMC group was more obvious than that in the Chronic Stress group and the T2DM group. BDNF and CaMK II were elevated in the CX3CR1 antibody intervention group.

Compared with the normal group, the model groups had a significant increase in CX3CR1 and FKN, which was even more obvious in T2DMC group. CX3CR1 and FKN expressions decreased after CX3CR1 intervention; in particular, the decrease of CX3CR1 expression was statistically significant (*P* < 0.01).

Compared with the normal group, the model groups had a significant increase in NR2A and NR2B. In the T2DMC group, the increase in the protein expressions of NR2A and NR2B was even more obvious than in the Chronic Stress group and the T2DM group. Compared with the model groups, the T2DMCC group had significantly decreased NR2A expression (Figures 7(b) and 7(d)).

The article "FKN/NR Signaling Pathway Regulates Hippocampal Inflammatory Responses: the Survival of Hippocampal Neurons in Diabetic Rats with Chronic Unpredictable Mild Stress" was published in 2022. Journal: Evid Based Complement Alternat Med.

### 3.9. Expression of CX3CR1, FKN, NR2A, and NR2B in Neuronal Cells under HCS Coculture System

HCS results showed that the expression of CX3CR1 fluorescent protein increased in cocultured hippocampal neurons compared with the normal group. The T2DMCC group was the lowest, indicating that the inhibitory effect of CX3CR1 neutralizing antibody was obvious. Compared with the normal group, the expression of FKN fluorescent protein increased in cocultured hippocampal neurons. FKN fluorescence expression increased in CX3CR1 group. Compared with the normal group, the expression of NR2A fluorescent protein increased in cocultured hippocampal neurons. NR2A expression can be regulated. At the same time, CX3CR1 can affect the expression of NR2A (Figure 8).

## 4. Discussion

Depression is one of the common complications of diabetes. Patients with diabetes mellitus with depression can increase their mortality and morbidity. The suicide rate in DD patients reaches 10% [21]. Hippocampus, especially CA1 region, is closely related to cognitive function and is an important organ involved with learning and memory [22–24].

Diabetic patients are prone to cognitive decline, mainly characterized by impaired hippocampal function. Hippocampal neuronal dysfunction can lead to depression. As an important excitatory amino acid receptor in the central nervous system, NR regulates the survival of hippocampal neurons [22, 25]. Microglia has neuroprotective capacities, yet chronic activation can promote neurotoxic inflammation. Neuronal fractalkine (FKN), acting on CX (3) CR1, has been shown to suppress excessive microglia activation.

FKN and CX3CR1 increase may cause a cross-talk between activated glial cells and neurons [26]. FKN/CX3CR1 plays an important role in the development of neuroinflammation and neuronal damage in hippocampus. FKN/CX (3) CR1 signaling in young adult rodents decreased survival and proliferation of neural progenitor cells through IL-1*β* [27], also leading to the reduction of proinflammatory cytokines TNF-*α* and IL-6 [28].

The MWM is widely used for the functional evaluation of brain regions related to spatial learning and memory and the open field test is a simple method to assess the locomotor activity of rats based on their innate tendency to avoid open spaces [29]. Both of them are important tools for evaluating depression-like behaviors in rodents. In the present study, open field test showed that the frequency of spontaneous activities decreased significantly in the Chronic Stress group and T2DMC group, along with markedly declined learning and memory abilities [30]. The CX3CR1 neutral antibody can be used to interfere with CX3CR1 secretion and acts as a CX3CR1 blocker [31]. In our study, the T2DMCC group showed both significantly increased spontaneous activity and significantly improved learning and memory abilities. DD rats had obvious depressive symptoms, which were alleviated after CX3CR1 antibody intervention, suggesting that the depression behaviors were affected by CX3CR1-related pathways in DD rats. In addition, the blood glucose level showed no significant change in the Chronic Stress group and the normal group, and the body weight gain was normal. In contrast, the average blood glucose levels in the T2DMC group and the T2DM group were significantly higher than those of other groups, along with markedly decreased body weight. The T2DMCC group had lower blood glucose and increased body weight. Thus, the blood glucose level was regulated by CX3CR1-related pathways in the diabetes models and T2DMC group.

The article "FKN/NR Signaling Pathway Regulates Hippocampal Inflammatory Responses: the Survival of Hippocampal Neurons in Diabetic Rats with Chronic Unpredictable Mild Stress" was published in 2022. Journal: Evid Based Complement Alternat Med.

The immune-inflammatory response plays a key role in the pathogenesis of depression and diabetes [32]. Studies have shown that diabetic patients complicated with depression have higher levels of inflammatory factors than normal subjects [33]. In our study, ELISA showed that the levels of three inflammatory factors significantly increased in each model group when compared with the normal group and the T2DMC group had the highest levels of inflammatory factors. Compared with the T2DMC group, the T2DMCC group showed a significant decrease in inflammatory factor levels. Therefore, the inflammatory factors are elevated under a DD state, whereas the CX3CR1 pathway may improve their levels. Glu is an excitatory neurotransmitter that plays an important role in maintaining the normal functional activities of the central nervous system and in regulating nerves [34]. However, high-concentration glutamate has neurotoxic effects and can damage neurons and thus induce neuropsychiatric diseases [35]. D-serine is an endogenous transmitter of the N-methyl-D-aspartic acid receptor in the central nervous system [36].

In our study, Glu and D-serine increased significantly in each model group. In addition, pathology showed that hippocampal injury was more severe in Chronic Stress group than in T2DM group and was even worse in T2DMC group. The Glu and D-serine levels decreased significantly after CX3CR1 antibody intervention, and the pathological state of hippocampus was relieved. Thus, the CX3CR1 signaling pathway can affect the secretion of neurotransmitters.

We found that the expression levels of BDNF, CaMK II, A1R, and A3R in hippocampus decreased in each model group, whereas the expression levels of A2R, CX3CR1, FKN, NR2A, and NR2B increased. After intervention with CX3CR1 antibody, the expressions of BDNF, CaMK II, A1R, and A3R increased and those of A2R, CX3CR1, FKN, NR2A, and NR2B decreased. Studies have shown that, at a diabetic state, the persistent hyperglycemia leads to increased expressions of inflammatory cytokines in the body [37]. After these inflammatory cytokines enter the brain through the damaged blood-brain barrier, the hippocampus can release excitatory neurotransmitters such as Glu, leading to neuronal injury [38]. Inflammatory cytokines in the brain can also cause a dramatic decrease in the secretion of neurotrophic factors such as brain-derived neurotrophic factor (BDNF), thereby attenuating the neuroprotective effect [39]. FKN, an effective neuromodulator for inducing excitatory synaptic transmission, can exert its effect by binding to its receptor CX3CR1 [40]. It has been reported that inflammatory factors can induce the abnormal neuronal secretion of FKN in diabetic or depressed patients [41]. The binding of FKN to its receptor CX3CR1 increases intracellular secretion of adenosine, which binds to its receptor and presents key biological activities and pharmacological characteristics in the hippocampus [42]. We inferred that, under diabetic condition, (a) abnormal increase in A2AR density promotes the release of a large amount of D-serine, an endogenous ligand for NR, resulting in excessive activation of NR on neurons [43]; (b) adenosine binds to the A1R, which leads to decreased BDNF secretion and neurotrophic deficiency [44]; and (c) inhibition of the A3R on neuronal membrane induces NMDA channel opening and increases intracellular Ca^2+^ concentration, resulting in Ca^2+^/CaMKII-dependent inhibition [45]. Therefore, FKN can regulate the density changes of NR receptor subtypes NR2A and NR2B through the FKN/CX3CR1 signaling pathway, leading to NR activation and thus mediating the abnormal change of hippocampal neurons.

The article "FKN/NR Signaling Pathway Regulates Hippocampal Inflammatory Responses: the Survival of Hippocampal Neurons in Diabetic Rats with Chronic Unpredictable Mild Stress" was published in 2022. Journal: Evid Based Complement Alternat Med.

In conclusion, under diabetic condition, cytokines increase significantly in hippocampus, activating the inflammatory pathway and thus increasing the expression and secretion of the chemokine FKN. The increased FKN binds to its receptor CX3CR1 and promotes the release of intracellular adenosine. Adenosine can further act on neurons through its receptors, overactivating neurons and leading to neuronal damage. Intervention with CX3CR1 neutral antibody can alleviate the neuronal damage.

The purpose of Morris water maze is to test the capability of learning and memory by place navigation and space exploration. As shown by MWM, the T2DMC model group had longer escape latency (EL) and was significantly lower in space exploration time (SET) when compared with normal group. Compared with the normal group, the learning and memory abilities of DD rats were significantly weakened while there were significant improvements in the T2DMCC group (*P* < 0.05 or *P* < 0.01) (Figure 2(a)).

In the OF, the horizontal activity and vertical activity were observed to evaluate the motion activity and curiosity in an open field. The result indicates that there was a downregulation in both Chronic Stress group and T2DMC group (*P* < 0.01). Otherwise, the total activity scores of horizon activities and vertical activities were significantly increased in the T2DMCC group (*P* < 0.05) (Figure 2(b)).

### 4.1. Effect of DD on Body Weight and Glucose in Diabetic Rats

The body weight of the rats was examined starting from the successful modeling (day 17 of the experiment). The body weight of the Chronic Stress group and the normal group increased with the stress modeling time. Starting from 31 days, rats in the T2DM group and T2DMC group were significantly thinner and their body weight decreased. However, the T2DMCC group showed significant weight gain during the last week of the experiment (Figure 2(c)).

### 4.2. The Blood Glucose Level of DD

The blood glucose level was measured every week. The blood glucose level showed no significant change in the Chronic Stress group and the normal group while the average blood glucose levels in the T2DMC group and the T2DM group were significantly higher than those of other groups. The blood glucose level decreased significantly in the T2DMCC group, suggesting that blocking the CX3CR1 signaling pathway had an effect on blood glucose (Figure 2(d)).

## Figures and Tables

**Figure 1:** Experimental timeline.

**Figure 2:** Abnormal body weight, blood glucose, and depressive-like behavior in DD rats. (a) The time of escape latency and space exploration for cognitive function of model rats. (b) The locomotion in open field. (c) Body weight. (d) Oral glucose tolerance test. (e) Number of activities in the open field test and the immobility time in the forced swimming test. Compared with the normal control group ^Δ^*P* < 0.05 and ^ΔΔ^*P* < 0.01; compared with the diabetes group, ^*∗*^*P* < 0.05 and ^*∗∗*^*P* < 0.01; compared with the depression group, ^#^*P* < 0.05 and ^##^*P* < 0.01; compared with the DD group, ^*P* < 0.05 and ^^*P* < 0.05.

**Figure 3:** Changes of insulin and glycosylated hemoglobin content of DD. Compared with the normal group ^Δ^*P* < 0.05 and ^ΔΔ^*P* < 0.01; compared with the diabetes group, ^*∗*^*P* < 0.05 and ^*∗∗*^*P* < 0.01; compared with the depression group, ^#^*P* < 0.05 and ^##^*P* < 0.01; compared with the DD group, ^*P* < 0.05 and ^^*P* < 0.01.

**Figure 4:** Compared with the normal group in information factor and Glu, D-serine levels, ^Δ^*P* < 0.05 and ^ΔΔ^*P* < 0.01; compared with the diabetes group, ^*∗*^*P* < 0.05 and ^*∗∗*^*P* < 0.01; compared with the diabetes group, ^#^*P* < 0.05 and ^##^*P* < 0.01; compared with the DD group, ^*P* < 0.05 and ^^*P* < 0.01.

The article "FKN/NR Signaling Pathway Regulates Hippocampal Inflammatory Responses: the Survival of Hippocampal Neurons in Diabetic Rats with Chronic Unpredictable Mild Stress" was published in 2022. Journal: Evid Based Complement Alternat Med.

**Figure 5:** Changes of monoamine neurotransmitters in hippocampus: ^Δ^*P* < 0.05 and ^ΔΔ^*P* < 0.01; compared with the diabetes group, ^*∗*^*P* < 0.05 and ^*∗∗*^*P* < 0.01; compared with the diabetes group, ^#^*P* < 0.05 and ^##^*P* < 0.01; compared with the DD group, ^*P* < 0.05 and ^^*P* < 0.01.

**Figure 6:** Findings of HE staining. (a) Normal group; (b) diabetic group; (c) depression group; (d) DD group; (e) DD + CX3CR1 antibody intervention group.

**Figure 7:** Immunohistochemical and Western-blotting of CX3CR1/FKN. (a) Immunohistochemical findings of CX3CR1/FKN-related molecules. (b) Western-blotting results of CX3CR1/FKN-related molecules. (c) Gray value of immunohistochemistry. (d) Gray value of Western-blotting. Compared with the normal control group, ^Δ^*P* < 0.05 and ^ΔΔ^*P* < 0.01; compared with the T2DM group, ^*∗*^*P* < 0.05 and ^*∗∗*^*P* < 0.01; compared with the T2DM group, ^#^*P* < 0.05 and ^##^*P* < 0.01; compared with the T2DMC group, ^*P* < 0.05 and ^^*P* < 0.01.

**Figure 8:** Expression of CX3CR1, FKN, NR2A, and NR2B in neuronal cells under HCS. (a) Expression picture in each group. (b) Comparison of protein expression of CX3CR1, FKN, NR2A, and NR2B in hippocampal neurons of each group under coculture. Note that, compared with the normal group, ^#^*P* < 0.05 and ^##^*P* < 0.01; compared with the model group, ^*∗*^*P* < 0.05 and ^*∗∗*^*P* < 0.01.

**Table 1:** 

	NA	DA	5-HT
Regression equation	*y* = 1333*x*^2^ − 5733*x* + 6019	*y* = 7415*x*^2^ − 29914*x* + 29853	*y* = 23.18*x*^2^ − 37.75*x* + 41.70
*r * ^2^	*R * ^2^ = 0.990	0.993	0.991

Standard curve of Na, Da, and 5-HT.

## Data Availability

The data used to support the findings of this study are available from the corresponding author upon request.

## Additional Points

*Possible Limitation of the Research*. An apparent limitation of the method is that it is an animal experiment, not a clinical sample. It can be further verified by clinical trials.
